RETRACTED

# Inhibiting of Proliferation, Migration, and Invasion in Lung Cancer Induced by Silencing Interferon-Induced Transmembrane Protein 1 (IFITM1)

**DOI:** 10.1155/2019/9085435

**Published:** 2019-05-08

**Authors:** Jun Yan, Ying Jiang, Jianfeng Lu, Jianhui Wu, Mingfang Zhang

**Affiliations:** Department of Pathology, Tianjin First Center Hospital, Tianjin 300192, China

## Abstract

Interferon-induced transmembrane protein 1 (IFITM1), a 17-kDa membrane protein, is generally known as a modulator in many cellular functions. Recent studies showed overexpression of IFITM1 in cancers and relationship between IFITM1 overexpression and tumor progression. However, the role of IFITM1 in lung cancer remains unclear. Here, we presented the overexpression of IFITM1 in lung cancer tissues and cell lines A549 and H460 using quantitative Real-Time RT-PCR.* In vitro *assay indicated IFITM1 silencing inhibited lung cancer cell proliferation, migration, and invasion. Further,* in vivo *assay showed that IFITM1 silencing markedly suppressed cell growth and metastasis of lung cancer in tumor-bearing BALB/c nude mice. Mechanistically, we found that IFITM1 silencing significantly alleviated the protein levels of *β*-catenin, cyclin D1, and c-Mycin lung cancer cells and tumor samples. Taken together, our study revealed the role of IFITM1 as a tumor promoter during lung cancer development and the possible molecular mechanism.

## 1. Introduction

Lung cancer, a common type of cancers in the world, is divided into two categories: small cell lung cancer (SCLC) and non-small-cell lung cancer (NSCLC) [1]. The latter accounts for about 80% of cases of lung cancer and is further classified into adenocarcinoma, squamous cell carcinoma, large cell carcinoma, and so on [2]. By far, therapeutic approaches for lung cancer include palliative care, surgery, radiation therapy, chemotherapy, and target therapy [3–5]. Despite a great improvement in these therapies, lung cancer still has a high mortality owing to late diagnosis and poor response to therapies [6, 7]. On the one hand, we shall explore potential markers to improve the diagnosis of lung cancer. On the other hand, we shall study the mechanisms underlying the progression of lung cancer to help make the treatment more effective.

Interferon-induced transmembrane protein 1 (IFITM1), a 17-kDa membrane protein, is part of membrane complexes transducing homotypic adhesion signals in lymphocytes [8–10]. It was originally identified as Leu13, a cell-surface membrane protein encoded on the short arm of chromosome 11[11–14]. Its expression is induced by IFN-*α* and, to a lesser extent, by IFN-*γ* and has been found in Jurkat cells, U937 cells, and K562 cells [15, 16]. IFITM1 is largely known as a player in many cellular functions such as adhesion and proliferation [17]. It is also important for immunity and antiviral activity [18]. In addition, IFITM1 has been reported to be related to inflammatory bowel disease, osteogenesis, and angiogenesis [19–21]. Recently, there have been studies showing overexpression of IFITM1 in some types of cancers such as gastrointestinal, colorectal, and breast cancers [22, 23]. Furthermore, these studies have demonstrated a positive correlation of IFITM1 overexpression with tumor progression. However, it is poorly understood what role IFITM1 plays in lung cancer.

RETRACTED

In this study, we presented evidence that IFITM1 was highly expressed in lung cancer tissues and cell lines. IFITM1 silencing inhibited lung cancer cell proliferation, migration, and invasion* in vitro*. Furthermore, the* in vivo* experiments showed that IFITM1 silencing inhibited lung cancer cell growth and metastasis. We also found that IFITM1 silencing decreased the protein levels of *β*-catenin, cyclin D1, and c-Myc. Taken together, our study suggested that IFITM1 might function as a tumor promoter during lung cancer development.

## 2. Materials and Methods

### 2.1. Patients and Tissue Samples

Lung cancer tissues and matching normal lung tissues were collected from 30 patients hospitalized at Tianjin First Center Hospital (Tianjin, China). No patients had received any adjuvant therapies before surgery. Each patient taking part in the study provided written consent. All tissues were frozen in liquid nitrogen and stored at -80°C until use. The study was approved by the Ethics Committee of Nanjing Medical University.

### 2.2. Cell Lines and Cell Culture

Human lung cancer cells (A549 and H460) and bronchial epithelial cells (BEAS-2B) were obtained from FuHeng Cell Center (Shanghai, China). All cell lines were cultured in RPMI 1640 (Sigma, St. Louis, MO, USA) containing 10% fetal bovine serum (FBS; Sigma) and 1% streptomycin/penicillin, followed by incubation at 37°C in a humidified atmosphere with 5% CO_2_.

### 2.3. Quantitative Real-Time RT-PCR

Total RNA was isolated from tissues or cells using TRIzol reagent (Invitrogen, Carlsbad, CA, USA) and then used for cDNA synthesis. Quantitative RT-PCR was carried out using Platinum SYBR Green qPCR SuperMix-UDG (Invitrogen). All reactions were performed in triplicate. The primers were listed as follows: IFITM1, 5'-ATGTCGTCTGGTCCCTGTTC-3' (forward) and 5'-GTCATGAGGATGCCCAGAAT-3' (reverse); GAPDH, 5'-TCCACCACCCTGTTGCTGTA-3' (forward) and 5'-ACCACAGTCCATGCCATCAC-3' (reverse). GAPDH was used as internal control. The 2^-ΔΔCt^ method was used to calculate the expression changes.

RETRACTED

### 2.4. Western Blot Analysis

Tissues or cells were lysed with ice-cold lysis buffer. Proteins were fractionated by 12% SDS-PAGE and then transferred onto PVDF membranes. After blocking in 5% skim milk, the membranes were probed with primary antibodies against IFITM1, *β*-catenin, cyclin D1, c-Myc, and GAPDH (Invitrogen). Subsequently, the membranes were washed three times with TBST buffer and then incubated at 4°C with appropriate secondary antibodies (Invitrogen). The proteins were detected using enhanced chemiluminescence (Millipore, Bredford, MA, USA). Immunoreactive bands were quantified with the Image J software.

### 2.5. Small Interfering RNA (siRNA) and Cell Transfection

The siRNA targeting human IFITM1 mRNA (si-IFITM1: 5'-AACTCATGACCATTGGATTCA-3') and a nonspecific scramble siRNA (si-Control: 5'-AACGTACGCGGAATACTTCGA-3') were synthesized and purified by Sigma-Proligo (Woodlands, TX, USA). These siRNAs were transiently transfected into A549 and H460 cells using Lipofectamine 2000 (Invitrogen) according to the manufacturer's instruction. The transfection efficiency was determined using western blot analysis.

### 2.6. MTT Assay

Cell proliferation was determined using MTT assay. In brief, cells were seeded into 96-well plates at a density of 2×10^3^ cells/well. MTT solution (5 mg/mL) was added to each well at indicated time and cells were incubated at 37°C for 4 h. After culture medium was removed, DMSO was added to each well. The optical density was read at 570 nm with a microplate reader.

### 2.7. Wound-Healing Assay

The migratory capability of lung cancer cells was examined using wound-healing assay. Briefly, cells were seeded in 6-well plates and grown to full confluency, followed by overnight incubation in starvation medium. Cell monolayer was scratched with a 10 *μ*L sterile pipette tip, washed with PBS, and then cultured in serum-free medium for 24h. Wound gaps were observed under Olympus BX41 microscope and photographed using a Qcolor5 digital camera.

### 2.8. Transwell Assay

Cell invasion was detected using transwell chambers with Matrigel-coated inserts (8*μ*m pore). 5×10^4^ cells in 200 *μ*L of serum-free medium were added to the upper chamber. 500 *μ*L of DMEM containing 10% FBS was added to the low chamber. After 24 h, cells remaining on the upper side of the insert were removed while those invading to the lower side were stained with 0.2% crystal violet. The number of invading cells was counted using a microscope.

### 2.9. Xenograft Tumor Assay

Male BALB/c nude mice (5 weeks old) were purchased from Shanghai Laboratory Animals Center (Shanghai, China) and used for xenograft experiments. All animal experiments were performed with the approval of the Ethics Committee of Nanjing Medical University. For tumorigenesis experiments, 2×106A549 cells transfected with si-IFITM1 or si-Control were resuspended in 0.1 mL PBS and subcutaneously injected into the right flank of nude mice (n = 6) and the mice were daily intratumoral injection of si-IFITM1 and si-Control for 35 days. The tumor size was measured every 7 days. After 35 days, mice were euthanized and tumors were resected and weighed. For metastasis experiments, 2×106 transfected A549 cells in 0.1 mL PBS were intravenously injected into the tail of nude mice (n = 6). 35 days later, mice were euthanized and metastasis nodules in lungs were counted.

RETRACTED

### 2.10. Statistical Analysis

Data from three independent experiments were shown as means ± standard deviation (SD). Statistical analysis was performed via SPSS 16.0 software. Comparisons between different groups were made using the Student's* t*-test.* P*< 0.05 was considered statistically significant.

## 3. Results

### 3.1. IFITM1Is Highly Expressed in Lung Cancer Tissues and Cell Lines

Before exploration of the role of IFITM1 in lung cancer, we examined its expression in lung cancer tissues and corresponding normal lung tissues using RT-PCR and western blot analysis. As shown in Figures 1(a) and 1(b), the mRNA and protein levels of IFITM1 were higher in lung cancer tissues than in the normal lung tissues. We also detected the expression of IFITM1 in two lung cancer cell lines (A549 and H460) and a bronchial epithelial cell line (BEAS-2B). The results showed that all lung cancer cell lines expressed higher mRNA and protein levels of IFITM1 in comparison with the BEAS-2B cell line (Figures 1(c) and 1(d)).

### 3.2. IFITM1 Silencing Inhibits Lung Cancer Cell Proliferation

In order to silence IFITM1, we transfected si-IFITM1 into A549 and H460 cells. The efficiency of IFITM1 silencing was examined by western blot. As shown in Figures 2(a) and 2(b), the protein levels of IFITM1 were markedly decreased in A549 and H460 cells after transfection with si-IFITM1.

Next, we determined whether IFITM1 silencing affected the lung cancer cell proliferation. For this purpose, we performed MTT assay. The results showed that IFITM1 silencing remarkably inhibited the proliferation of A549 and H460 cells (Figures 2(c) and 2(d)). In addition, cell cycle progression of A549 and H460 cells was slowed down in IFITM1 silenced cells (Figures 2(e) and 2(f)).

### 3.3. IFITM1 Silencing Inhibits Lung Cancer Cell Migration and Invasion

To investigate the effect of IFITM1 silencing on lung cancer cell migration, the wound-healing assay was performed. In both A549 and H460 cells, IFITM1 silencing significantly inhibited the wound-healing process, indicating a decreased cell migration induced by IFITM1 silencing (Figures 3(a) and 3(b)). We further examined the function of IFITM1 silencing in the invasive capability of lung cancer cells. As shown by the transwell assay, the number of invading A549 and H460 cells was greatly reduced after IFITM1 silencing in comparison with the control cells (Figures 3(c) and 3(d)).

RETRACTED

### 3.4. IFITM1 Silencing Inhibits Lung Cancer Cell Growth and Metastasis In Vivo

We examined the* in vivo* tumorigenesis effect of IFITM1 silencing via subcutaneous injection of A549 cells into nude mice. Every 7 days, the tumor size was measured. 35 days later, mice were euthanized and tumors were weighed. The results showed that tumor volume and tumor mass were significantly reduced by IFITM1 silencing in comparison with the control group (Figures 4(a) and 4(b)). In metastasis experiments, we intravenously injected si-IFITM1-transfected A549 cells or control cells into nude mice. 35 days later, mice were euthanized to check for lung metastasis. The results indicated a remarkable decrease in the number of metastasis nodules in lungs (Figure 4(c)). The western blot assay revealed that the protein levels of *β*-catenin and its downstream targets cyclin D1 and c-Myc in tumor samples were significantly lower than that in control group (Figure 4(d)).

### 3.5. IFITM1 Silencing Inhibits the Activity of Wnt/*β*-Catenin Signaling Pathway

To investigate the underlying mechanisms by which IFITM1 played its role in lung cancer development, we examined the effect of IFITM1 silencing on the activity of Wnt/*β*-catenin signaling pathway which has been reported to be closely related to IFITM1[23, 24]. As shown in Figure 5, IFITM1 silencing significantly decreased the protein levels of *β*-catenin and its downstream targets cyclin D1 and c-Myc in A549 cells compared with the control cells, suggesting an inhibitory effect of IFITM1 silencing on the Wnt/*β*-catenin signaling pathway.

## 4. Discussion

With a steadily rising incidence in the world, lung cancer is a leading cause of cancer-related death. According to statistics, more than 1 million people die of lung cancer every year and this number continues to rise [25]. Such situation has attracted worldwide attention. With medical development, many potential markers for prognosis of lung cancer have been found such as serum carcinoembryonic antigen, neuron specific enolase, cytokeratin fragment, tissue polypeptide specific antigen, and progastrin-releasing peptide [26–28]. But their clinical values are limited due to their low specificity and sensitivity. So it is necessary to explore new special markers for improvement in the diagnosis of lung cancer.

RETRACTED

IFITM1, an encoder of secretary or cell-surface proteins involved in cell adhesion, angiogenesis, and growth factor, was recently reported to be a novel candidate for oncogenes [29]. For example, IFITM1 has been found overexpressed in esophageal cancer, colon cancer, ovarian cancer, and cervical cancer [22, 30–32]. In agreement with data obtained from the other cancer studies mentioned above, we measured the expression levels of IFITM1 in lung cancer tissues and cell lines. Our study results showed that IFITM1 was highly expressed in lung cancer tissues and cell lines. In the following experiments, we found that IFITM1 silencing inhibited lung cancer cell proliferation, migration, and invasion. These* in vitro *results were verified by our xenograft tumor assays which showed that IFITM1 silencing suppressed lung cancer cell growth and metastasis* in vivo*. More importantly,* Yang et al.* showed that IFITM1 was closely associated with a poor prognosis of non-small-cell cancer in patients; this was evidenced by a significantly low overall survive rate of IFITM1-positive patients versus IFITM1-negative patients [33]. However, it is still not clear how IFITM1 is induced in the lung cancer. Kim et al. reported that CD147 stimulation, which was implicated in tumor invasion, metastasis, and angiogenesis, could induce the expression of IFITM1 using a leukemic cell line [34]. Thus, we expect that unknown factors, which need to be explored further, may be enriched in lung cancer cell, and induce IFITM1 expression, could enhance tumor proliferation, invasion, and metastasis.

Consistently, Yu* et al*. reported that knockdown of IFITM1 had an inhibitory effect on the proliferation, migration, and invasion of glioma cells [35]. Other studies on IFITM1 provided further evidence for the oncogenic role of IFITM1. For instance, He* et al*. demonstrated that IFITM1 enhanced the invasive and metastatic capacity of colorectal cancer cells [36]. Hatano* et al*. found that IFITM1 promoted invasion during the progression of head and neck cancer [37]. These observations supported the idea that IFITM1 exerted an oncogenic function in cancer development.

It was documented that the cytoplasmic protein *β*-catenin served as the key switch in the Wnt pathway [38], and the perturbation of Wnt signaling could dramatically suppress lung tumor progression [39]. The Wnt/*β*-catenin signaling pathway takes part in modulation of some crucial cellular processes including proliferation, invasion, apoptosis, and differentiation [40–42]. More importantly, the Wnt/*β*-catenin signaling pathway has been found playing a significant role during lung cancer development. Previous studies on NSCLC demonstrated that the proliferation and migration of lung cancer could be inhibited by targeting the Wnt/*β*-catenin signaling pathway [43, 44]. Earlier studies have reported that the Wnt/*β*-catenin signaling is a controller of the expression levels of IFITM1 and that activation of the Wnt/*β*-catenin signaling may induce IFITM1 during intestinal tumorigenesis [23, 24]. To know the mechanism underlying the tumor-promotion role of IFITM1 in lung cancer cells, we investigated the effect of IFITM1 silencing on the Wnt/*β*-catenin signaling pathway. In this study, we observed that IFITM1 silencing significantly decreased the protein levels of *β*-catenin, cyclin D1, and c-Myc in lung cancer cells and tumor tissues, indicating an inhibitory effect of IFITM1 silencing on the Wnt/*β*-catenin signaling pathway. Based on all the results in our study, we suggested that IFITM1 silencing inhibited lung cancer progression, at least in part, via regulating the Wnt/*β*-catenin signaling pathway.

RETRACTED

In conclusion, our data demonstrated for the first time that IFITM1 was overexpressed in lung cancer tissues and cell lines. Silencing of IFITM1 inhibited proliferation, migration, and invasion of lung cancer cells. Furthermore, we found that IFITM1 silencing inhibited lung cancer cell growth and metastasis* in vivo*. We further showed that IFITM1 silencing had a suppressive effect on the Wnt/*β*-catenin signaling pathway. Taken together, our study suggested IFITM1 as a novel molecular target for treatment of lung cancer.

## Figures and Tables

**Figure 1:** *IFITM1 is highly expressed in lung cancer tissues and cell lines.* (a, b) RT-PCR and western blot analysis of IFITM1 expression in lung cancer tissues and matching normal lung tissues. (n=30). (c, d) RT-PCR and western blot analysis of IFITM1 expression in lung cancer cell lines (A549 and H460) and a bronchial epithelial cell line (BEAS-2B). *∗P*< 0.05.

**Figure 2:** *IFITM1 silencing inhibits lung cancer cell proliferation.* (a, b) IFITM1 silencing by siRNA notably reduced the protein expression levels of IFITM1 in A549 and H460 cells. (c, d) Cell proliferation was measured in si-IFITM1 or si-Control transfected A549 and H460 cells by MTT assay. (e, f) Cell cycle phase patterns of A549 and H460 cells. *∗P*< 0.05.

**Figure 3:** *IFITM1 silencing inhibits lung cancer cell migration and invasion.* (a, b) The wound-healing assay was performed to measure the effect of IFITM1 silencing on the migratory ability of A549 and H460 cells. (c, d) The transwell assay was performed to detect the effect of IFITM1 silencing on the invasive ability of A549 and H460 cells. *∗P*< 0.05.

RETRACTED

**Figure 4:** *IFITM1 silencing inhibits lung cancer cell growth and metastasis in vivo.* (a, b) The growth curve and weight of tumors from si-IFITM1-transfected A549 cells or control cells. (c) Quantification of metastasis nodules in lungs 35 days after intravenous injection of the transfected A549 cells or control cells. (d) Levels of *β*-catenin, cyclin D1, and c-Myc in tumor samples were detected by western blot. (n=6) *∗P*< 0.05.

**Figure 5:** *IFITM1 silencing inhibits the activity of Wnt/β-catenin signaling pathway.* (a) The western blot showed a significant decrease in the protein expression levels of *β*-catenin, cyclin D1, and c-Myc in si-IFITM1-transfected A549 cells compared with the control cells. (b) The relative protein expression levels of *β*-catenin, cyclin D1, and c-Mycin A549 cells were quantified by Image J software. *∗P*< 0.05.

## Data Availability

The data used to support the findings of this study are included within the article.
